# Meta-Analysis of the Effect of Aerobic Training on Blood Pressure in Hypertensive Patients

**DOI:** 10.1155/2022/9281661

**Published:** 2022-05-25

**Authors:** Yanping Fu, Qiongfang Feng, Yingna Wei, Liang Fan, Yandie Pan, Jingui Ji, Chengxia Lin

**Affiliations:** ^1^Department of Internal Medicine-Cardiovascular, Sanya Central Hospital (Hainan Third People's Hospital), Sanya, 572000 Hainan, China; ^2^Department of Emergency, Dongfang People's Hospital, Dongfang, 572600 Hainan, China; ^3^Outpatient Department, Haikou Hospital of Traditional Chinese Medicine, Haikou, 570216 Hainan, China; ^4^Department of Lung and Heart Disease, Haikou Hospital of Traditional Chinese Medicine, Haikou, 570216 Hainan, China

## Abstract

**Background:**

We aimed to evaluate the effect of different aerobic training methods and exercise duration on blood pressure in hypertensive patients, including systolic blood pressure (SBP) and diastolic blood pressure (DBP).

**Methods:**

Using the literature review method, the English database PubMed was retrieved to obtain relevant research literature, and the selected studies were analyzed and evaluated.

**Results:**

14 clinical studies were included in this study, with a total of 1027 patients, including 681 in the aerobic training group and 409 in the control group. Based on heterogeneity test results, the differences of SBP and DBP before and after the physical intervention were combined using a random effect model. The results indicated that the aerobic training group could significantly reduce SBP compared with the control group, WMD = −9.91, 95% CI (-14.21, -5.61), *P* < 0.0001. The DBP was reduced significantly in the aerobic training group, WMD = −4.32, 95% CI (- 7.02, -1.62), *P* < 0.001. The results of subgroup analysis showed that both progressive training and nonprogressive training could reduce blood pressure in patients, and training time less than 12 weeks and more than 12 weeks could reduce blood pressure in patients.

**Conclusion:**

Implementing aerobic training can effectively reduce blood pressure in hypertensive patients. Progressive training, nonprogressive training, and different training cycles can all benefit hypertensive patients.

## 1. Introduction

Hypertension, a multifactorial chronic disease, is one of the major health concerns which affects more than 1 billion adults worldwide [1]. The current percentages of people suffering from hypertension in China is 25.2% and increasing by years [2, 3]. As known, hypertension is closely related to several cardiovascular incidence and mortality rates. Thus, hypertension is identified as an important risk factor for vascular diseases [4, 5] and could bring severe diseases and financial burdens to families and society. Other than drug treatments, active lifestyle could significantly ameliorate hypertension syndrome as well [6].

In physical therapy, moderate-intensity aerobic exercise often supplemented with dynamic resistance training, as the first-class recommendation of the guide, is the main way to decrease blood pressure. A meta-analysis showed that moderate-intensity training had the best blood pressure improvement effect in hypertensive patients, while high-volume high-intensity interval training was more effective in reducing body weight and resting heart rate [6]. Off notes, aerobic exercise was considered a great starting point for hypertensive patients compared with moderate-intensity training and high-intensity training per antihypertensive physical therapy guidelines. Several review articles have concluded that aerobic exercise appeared to be beneficial in blood pressure control in patients with hypertension [7]. Different training variables, such as prior progressive training for patient adaptation, could affect the antihypertensive effect of aerobic training. Progressive training is defined as gradually or systematically increasing the training intensity, such as increasing the frequency and intensity of training with health improvement to promote continuous training adaptability [8]. In addition, the length of training also contributed to the training effects. With the significance in clinic, this study adopted the method of meta-analysis, including the latest research on the treatment of hypertension with aerobic training, to conduct a quantitative study on the antihypertensive effect of aerobic training. In brief, this study performed a subgroup analysis to analyze the impact of progressive training and the length of exercise on the antihypertensive effect.

## 2. Materials and Methods

### 2.1. Literature Retrieval Strategy

PubMed, an English database, was searched for published clinical trials on the effect of aerobic training on blood pressure in patients with hypertension from January 2010 to March 2022. The retrieval method was medical subject words combined with free words. The English retrieval subject words were “hypertension OR blood pressure high OR high blood pressure” AND “exercise OR physical exercise OR exercise aerobic OR aerobic exercise OR exercise training” AND “blood pressure OR diastolic pressure OR systolic pressure”. At the same time, the references were manually retrieved in the relevant literature.

### 2.2. Literature Screening

Inclusion criteria are as follows: (1) The subjects were adults with hypertension (≥ 18 years old) who participated in at least four weeks of supervision and structured aerobic exercise intervention. (2) The study should at least be a two-arm study, including at least the experimental group receiving aerobic training and the control group not receiving aerobic training. (3) The outcome index includes at least one of diastolic blood pressure (DBP) and systolic blood pressure (SBP), and the value of diastolic/systolic blood pressure before and after intervention or the difference before and after intervention can be obtained.

Exclusion criteria are as follows: (1) some or all patients in the study received other types of physical training in addition to aerobic training; (2) hypertensive patients with cardiovascular diseases such as heart failure, coronary artery disease, and peripheral artery disease; (3) news reports, expert opinions, critical literature, and abstracts; (4) duplicate published literature; (5) unbalanced baseline data between the experimental and control groups; and (6) unable to obtain enough literature to analyze the data.

### 2.3. Document Data Extraction

According to the above inclusion and exclusion criteria, two professional researchers independently screened the literature, determined the final included literature, and extracted the data according to the predetermined data extraction table. The main extraction contents include (1) basic information, including title, publication date, and author's name; (2) data included in the literature, including research type, research population, intervention measures, and outcome indicators; and (3) characteristics of included literature, including research methods, object characteristics, and data results. Suppose there are questions or differences in the process of literature screening and extraction. In that case, a third researcher will assist in resolving the differences and decide through discussion at the meeting if necessary.

### 2.4. Literature Quality Evaluation

The quality of the included literature was evaluated according to the risk bias evaluation tool in the Cochrane manual. The evaluation contents include (1) whether the random allocation method is appropriate, (2) whether the random allocation scheme is hidden, (3) whether the blind method is adopted, (4) whether the result data is complete, (5) whether there are selective reports of results, and (6) whether there are other sources of bias. The evaluation results were divided into high risk, low risk, and uncertain risk. Two researchers independently evaluated the quality of the included literature and then cross-checked it. If there is any difference, both researchers will discuss it to reach an agreement or rule by the third researcher.

### 2.5. Statistical Method

This study used Cochrane software RevMan5.4 statistical analysis of all data. Taking the weighted mean difference (WMD) and 95% CI as the effect quantity, the effects of aerobic training and no aerobic training on diastolic and systolic blood pressure in patients with hypertension were statistically described by combining with the mean value, standard deviation, and sample size of the difference between SBP and DBP at baseline and after the intervention. After using the fixed-effect model or random effect model, it was considered statistically significant when *P* < 0.05. The Chi-square test was used to test the heterogeneity between different studies. When the *I*^2^ corrected by degrees of freedom was more than 50%, it was considered to be heterogeneous, and the random effect model was used. When *I*^2^ corrected by degrees of freedom is ≤50%, it was considered no heterogeneity, and the fixed effect model was adopted. The potential publication bias was estimated by funnel plot.

## 3. Results

### 3.1. Literature Search Results

In this study, 4558 relevant literatures were obtained through database retrieval. After retrieval, all literature were duplicated by EndNote X9 and manually screened based on topics and abstracts topics and abstracts using preestablished inclusion and exclusion criteria. The prescreened literatures were then fully assessed basing on full text for final selection. In this study, there were 14 literatures fitted into all designed criteria and were included for final meta-analysis. The specific screening process and results are shown in Figure 1.

### 3.2. Basic Characteristics and Quality Evaluation of Literature

All 14 included studies were published as English literature. The summary of basic information for 14 included studies was shown in Table 1. As indicated earlier, the publication time ranged from 2010 to 2021. Thus, the included literatures were up to most possible current date. Overall, for this meta-analysis, both randomized controlled trials and observational studies were included. There were 1027 patients with hypertension in total, including 681 in the aerobic training group and 409 in the control group with no sexual bias, whose ages were all over 35 years old. In general, the durations of aerobic training were all over 4 weeks including 4 weeks for one study, 6 weeks for one study, 8 weeks for four studies, 12 weeks for six studies, and 20 weeks for one study. Aerobic exercise mainly included walking, running, swimming, cross-country, track and field, and cyclic dynamometer. In the aspect of progressive training, progressive training prior to aerobic training was adapted in 7 literatures while the others did not include progressive training period. The exercise duration was between 20 and 60 minutes, averaged at 40 min, which fell into the recommended exercise time frame by professional. The exercise frequency was three times a week. The difference of SBP and DBP between the aerobic training group and the control group after training were shown in Table 2. Taken from this table, the aerobic training showed some degree of beneficial effects in reducing blood pressure in patients with hypertension.

Cochrane risk bias evaluation tool was used to evaluate the included literature. Only three literatures fully adopted the principles of randomization, distributive concealment, and blind method, and the evaluation quality was low risk. Most of the other literatures did not describe randomization, distributive concealment, and blind method, and the quality of risk was uncertain.

### 3.3. Meta-Analysis Results

#### 3.3.1. Meta-Analysis Results

14 literatures have reported the effects of aerobic training on SBP and DBP in patients with hypertension. The heterogeneity test results *I*^2^ of the two outcome indicators were 99%, indicating high heterogeneity. Therefore, the random effect model was used to merge the data. The meta-analysis results showed that the decline values of SBP and DBP in the aerobic training group before and after physical intervention were significantly higher than those in the control group. The difference of SBP in the aerobic training group was 8.90 mmHg lower than that in the control group. The combined result was WMD = −8.90, 95% CI (- 13.19, - 4.61), *P* < 0.0001, as shown in Figure 2. The difference of SBP was 4.59 mmHg lower than that in the control group. The combined result was WMD = −4.59, 95% CI (-7.38, -1.79), *P* = 0.001, as shown in Figure 3.

The publication bias was also taken into consideration as there were more than 10 literatures included in this study. The results showed that the included literatures were not symmetrically distributed around the combined effect WMD value. The funnel of SBP difference results was shown in Figure 4, distributed in the upper right corner, and the funnel of DBP difference results was shown in Figure 5, distributed in the upper part of the set. Taken from the funnel evaluation, there was obvious publication bias introduced. To overcome the publication bias, further subgroup analysis of the results was conducted.

#### 3.3.2. Subgroup Analysis Results

The meta-analysis results suggested that there were apparent heterogeneity and publication bias. Therefore, subgroup analysis was conducted based on whether or not progressive training was performed and on the duration of training. We applied a 12-week cutoff based on the median training duration in the included literature. The subgroup analysis results indicated that the differences of SBP and DBP in the experimental group without progressive training and the training cycle ≤ 12 weeks after intervention were lower than those in the control group (*P* < 0.05). The differences were statistically significant (see Tables 3 and 4).

## 4. Discussion

This study reviewed the literature and meta-analysis of the effects of aerobic training on systolic and diastolic blood pressure in adult patients with hypertension. The main methods of aerobic training included in the literature were walking, running, swimming, cross-country, track and field, and cyclic dynamometer. The training intensity and frequency were gradually increased according to the adaptability of patients. This type of progressive training was approved to be beneficial on training effect to patients; however, it is uncertain whether progressive training has any impacts on SBP and DBP compared with conventional training. In addition, extended training duration did not cause further effects on blood pressure. Taken combined results and subgroup analysis together, in this study, aerobic training significantly reduced SBP and DBP compared with the control group.

The conclusion of this study is consistent with the published conclusion on the effect of aerobic training on blood pressure in patients with hypertension. The meta-analysis results of Cao et al. [7], Igarashi et al. [23], and de Barcelos et al. [24] illustrated the reduction of SBP and DBP in the aerobic training group were about 8-12 mmHg and 5-6 mmHg, respectively. In this study, the WMD of the difference before and after the intervention was used as the effect quantity. The difference before and after the intervention in the aerobic training group was 9.91 mmHg lower than that in the control group, and the DBP was 4.32 mmHg lower, which further confirmed the antihypertensive effect of aerobic training. A previous study has shown that blood pressure decrease in patients with hypertension has significant clinical significance. A 10 mmHg reduction in SBP could reduce the risk of cardiovascular disease by 20%, stroke by 27%, and death by 13% [25].

Exercise intensity, duration, and frequency of each exercise played roles in regulating exercise effects. Relevant guidelines recommend moderate-intensity aerobic exercise, 30 to 60 minutes a day or 150 minutes a week, with a frequency of 4 to 7 times a week for training patients with hypertension [26]. In addition, it is generally recommended to gradually increase the exercise intensity, duration, and frequency using a progressive training to improve the effect of aerobic exercise. This study conducted a subgroup analysis on the use of progressive training. The results showed that the SBP with progressive training decreased more than those without progressive training, and there was no difference found in DBP. Subgroup analysis of training duration showed that when the training time was less than 12 weeks, the decline of SBP in the aerobic training group was higher, but the decrease of DBP was lower.

In one word, this study further confirmed that aerobic training has a significant effect on reducing diastolic and systolic blood pressure in patients with hypertension. Whether to use progressive training or whether the training time is longer than 12 weeks played little role. Therefore, it is suggested to select appropriate exercise methods and duration according to the guideline's recommendations for regular training in patients with hypertension.

## Figures and Tables

**Figure 1:** Document screening process and results.

**Figure 2:** SBP difference between the aerobic training group and control group before and after intervention.

**Figure 3:** Forest diagram of DBP difference between the aerobic training group and control group before and after intervention.

**Figure 4:** Funnel chart of SBP difference between the aerobic training group and control group before.

**Figure 5:** Funnel chart of DBP difference between the aerobic training group and control group before and after intervention.

**Table 1:** Basic characteristics of included literature.

ID	Progressive training	Age	Training time	Training mode	Duration	Weekly frequency
Abdelaal and Mohamad 2015 [9]	Yes	52.5	12 weeks	Treadmill	Start:20-35 min end:40-50 min	3
Baghaiee et al. 2018 [10]	Yes	38.1	12 weeks	NR	Start:25 min end:45 min	3
Farahan et al. 2010 [11]	Yes	47.7	10 weeks	Aquatic sports	35 min	3
Lamina 2010 [12]	Yes	58.4	8 weeks	Cyclic dynamometer	Start:45 min end:60 min	3
Latosik et al. 2014 [13]	Yes	NR	8 weeks	Cross country walking	45 min	NR
Soltani et al. 2020 [14]	Yes	47.9	8 weeks	Walking/running	27 min	3
Wong et al. 2018 [15]	Yes	73.5	20 weeks	Swimming	Start:25-30 min end:40-45 min	3-4
Arca et al. 2014 [16]	No	64	12 weeks	Cyclic dynamometer aquatic sports	20 min	3
Blumenthal et al. 2021 [17]	No	63	4 weeks	NR	30-40 min	3
He et al. 2018 [18]	No	57.5	12 weeks	Walking	60 min	3
Khalid et al. 2013 [19]	No	52.8	8 weeks	Walking	20 min	3
Izadi et al. 2018 [20]	No	61.6	6 weeks	Cyclic dynamometer	35 min	3
Maruf et al. 2014 [21]	No	52.0	12 weeks	Dancing	35 min	3
Ramos et al. 2018 [22]	No	60.6	12 weeks	Athletics	50 min	3

**Table 2:** Results of blood pressure difference between SBP and DBP included in the literature.

ID	Sample		SBP				DBP			
			Aerobic training group		Control		Aerobic training group		Control	
	Experimental group	Control group	Mean	sd	Mean	sd	Mean	sd	Mean	sd
Abdelaal et al. 2015 [9]	20	19	-4.95	2.50	0.68	3.20	-4.20	1.30	0.58	1.71
Baghaiee et al. 2018 [10]	20	20	-0.56	0.26	0.04	0.25	-0.01	0.49	0.02	0.05
Farahani et al. 2010 [11]	12	28	-16.67	12.16	-1.78	11.35	-4.17	90.54	0.18	6.49
Lamina 2010 [12]	252	105	-14.99	16.64	2.60	16.18	-4.25	7.98	-1.07	2.62
Latosik et al. 2014 [13]	15	10	-10.20	13.18	-6.60	6.00	-2.00	8.33	-0.60	4.01
Soltani et al. 2020 [14]	20	10	-8.00	13.69	2.00	11.27	-6.50	11.75	1.00	5.92
Wong et al. 2018 [15]	52	48	-11.00	1.18	1.00	1.18	-9.00	1.18	0.00	1.18
Arca et al. 2014 [16]	33	14	-12.00	16.73	-1.00	2.37	-8.00	1.31	-4.00	1.18
Blumenthal et al. 2021 [17]	90	50	-12.20	11.83	-7.20	11.83	-5.80	10.65	-4.40	9.47
He et al. 2018 [18]	20	22	-8.30	6.28	2.20	5.48	-1.10	5.11	0.80	3.83
Khalid et al. 2013 [19]	12	13	-24.00	6.63	-9.00	7.93	-9.00	5.72	0.00	4.69
Izadi et al. 2018 [20]	15	15	-3.43	7.73	0.67	7.40	-2.13	4.33	0.93	4.90
Maruf et al. 2014 [21]	45	43	-18.77	15.65	-8.81	18.84	-8.98	11.78	-5.60	12.72
Ramos et al. 2018 [22]	12	12	−4.4	5.20	6.10	3.50	-10.10	3.30	1.30	3.40

**Table 3:** Subgroup analysis of the effect of aerobic training on SBP.

Variables	Number of literatures (articles)	Heterogeneity test		Effect magnitude		
		*I* ^2^ value	*P* value	WMD value	95% CI value	*P* value
Progressive training						
Yes	7	100	<0.001	-9.07	(-15.25, -2.89)	<0.001
No	7	54	0.03	-8.18	(-10.87, -5.5)	<0.001
Training cycle						
<12 weeks	7	82	<0.001	-10.08	(-15.14, -5.02)	<0.001
≥12 weeks	7	100	<0.001	-7.35	(-12.98, -1.71)	0.01

**Table 4:** Subgroup analysis of the effect of aerobic training on DBP.

Variables	Number of literatures (articles)	Heterogeneity test		Effect magnitude		
		*I* ^2^ value	*P* value	WMD	*I* ^2^ value	*P* value
Progressive training						
Yes	7	100	<0.001	-4.26	(-8.75, 0.24)	0.06
No	7	83	<0.001	-4.45	(-6.86, -2.04)	<0.001
Training cycle						
<12 weeks	7	45	0.09	-3.37	(-4.32, -2.43)	<0.001
≥12 weeks	7	99	<0.001	-4.44	(-8.16, -0.73)	0.02

## Data Availability

The data used to support the findings of this study are included within the article.
